# Evaluation of Inflammatory Infiltration in the Retroperitoneal Space of Acute Pancreatitis Using Computer Tomography and Its Correlation with Clinical Severity

**DOI:** 10.1155/2023/7492293

**Published:** 2023-04-18

**Authors:** YuLong Xu, ChunJuan Ye, Bing Tan

**Affiliations:** Department of Emergency Medicine, Anhui No. 2 Provincial People's Hospital, Hefei 230041, Anhui, China

## Abstract

This paper investigates the correlation between the degree and severity of CT inflammatory infiltration in the retroperitoneal space of acute pancreatitis (AP). A total of 113 patients were included based on diagnostic criteria. The general data of the patients and the relationship between the computed tomography severity index (CTSI) and pleural effusion (PE), involvement, degree of inflammatory infiltration of retroperitoneal space (RPS), number of peripancreatic effusion sites, and degree of pancreatic necrosis on contrast-enhanced CT at different times were studied. The results showed that the mean age of onset in females was later than that in males; 62 cases involved RPS to varying degrees, with a positive rate of 54.9% (62/113), and the total involvement rates of only the anterior pararenal space (APS); both APS and perirenal space (PS); and APS, PS, and posterior pararenal space (PPS) were 46.9% (53/113), 53.1% (60/113), and 17.7% (20/113), respectively. The degree of inflammatory infiltration in the RPS worsened with the increase in CTSI score; the incidence of PE was higher in the group greater than 48 hours than in the group less than 48 hours; necrosis >50% grade was predominant (43.2%) 5 to 6 days after onset, with a higher detection rate than other time periods (*P* < 0.05). Thus, when the PPS was involved, the patient's condition can be treated as severe acute pancreatitis (SAP); the higher the degree of inflammatory infiltration in the retroperitoneum, the higher the severity of AP. Enhanced CT examination 5 to 6 days after onset in patients with AP revealed the greatest extent of pancreatic necrosis.

## 1. Introduction

Acute pancreatitis (AP) is caused by the early activation of many lytic enzymes (such as pancreatic lipase and trypsin) in the pancreas under the influence of various causes of the disease, resulting in different “autolytic” destruction of pancreatic acinar cells, pancreatic ductal epithelial cells, and pancreatic cells, and pancreatic edema, massive hemorrhage, and pancreatic/peripancreatic necrosis can be observed [1, 2]. In China, AP is a common and frequently occurring disease of the human digestive system, but due to different severities, many occurrences, and high mortality rates, AP has become a “challenging” serious acute abdomen disease that seriously affects the health of the Chinese people. AP, as a heterogeneous condition, has numerous causes and is divided into congenital causes and acquired causes [3]. Congenital factors are mainly divided into hereditary genetic causes, changes in pancreaticobiliary development/changes in pancreaticobiliary junction, pancreatic division, and annular pancreas. In addition, because AP is a systemic disease, it often leads to pathophysiological changes in many organ systems of the body, which can produce systemic complications and local complications in both the early and late stages of the disease [4]. After the diagnosis of AP, physicians must evaluate the severity of the patient's disease, but the prognosis of patients with AP of different severities is completely different. From the historical record of AP, there are various ways and related studies to diagnose the severity of the disease. Usually, clinicians try to determine the patient's condition by obtaining an indicator or some indicator in the patient's plasma sample by means of blood examination, while imaging scientists have to determine the patient's condition through the patient's imaging test data [5, 6]. At present, the diagnosis of AP can be roughly judged based on abdominal pain findings and imaging diagnosis, but the classification of its severity and the judgment of pancreatic necrosis are not deep enough.

AP is a systemic disease in which, in addition to a peripancreatic leak, extravasation of inflammatory cells can spread through many retroperitoneal spaces (RPS), intermediate levels of fascia, subperitoneal spaces, and the abdominopelvic cavity with extensive involvement [7]. Studies have confirmed that the infiltration thickness of left subphrenic fat presents a significant positive correlation with both the Ranson score and Balthazar grade, which can reflect the severity of clinical research conditions to some extent [8–10]. Inflammatory effusions resulting from peripancreatic/extrapancreatic exudates may propagate into many spaces in the body, including the APS, omental bursa, and intraperitoneal spaces in the abdominopelvic cavity that are of interest to the radiologists. However, other common anatomical sites are likely to be overlooked in daily work, such as the subperitoneal space and gastric bare area and the left subphrenic extraperitoneal space [11, 12]. The anterior layer of the right anterior renal fascia runs to the left at the front edge of the horizontal descending segment of the duodenum, and the posterior layer at the posterior edge of the descending segment of the duodenum continues to extend to the connective tissue membrane near the inferior vena cava to the left. Therefore, the bilateral anterior renal fascia running inward at the connective tissue membrane segment of the anterior inferior vena cava forms the extension of the same fascial layer, while the inflammatory effusion layer extends along the interfascial pathway, resulting in the consistency of both sides. This anatomical basis can explain the continuous imaging findings of CT/MRI images of bilateral APS effusion in front of the retroperitoneal great vessels (inferior vena cava and abdominal aorta), and it is speculated that this anatomical basis may also be one of the mechanisms of AP patients with bilateral APS effusion often coexisting. Most researchers have proposed that AP continues to spread to the RPS, including pancreatic enzyme infiltration rich in AP, which can cause the dissolution of renal fascia and inflammatory edema and effusion between renal fascia due to the histolytic effect. When the inflammation exceeds the prerenal and retrorenal fascia, the inflammation continues to proliferate and infiltrate the APS, PS, and PPS, causing transfascial and interspace diffusion of retroperitoneal changes [13].

The diagnosis and classification of pathology is a commonly used “gold standard” in clinical practice. For AP, it is difficult to obtain pancreatic and peripancreatic histological samples for medical data analysis because general patients do not undergo postoperative treatment and puncture angiographic sections during hospitalization [14]. Therefore, the current “gold standard” for the treatment of AP is to perform ultrasound imaging examination, generally enhanced CT examination. The CTSI scoring modality also has an important impact on predicting the severity of pancreatitis [15, 16]. CT examination is also helpful for diagnosis, and evaluation of the severity of the disease, such as pancreatic enlargement, decreased pressure, slurred contour, and peripancreatic exudate, can be observed during plain CT, while enhanced CT examination is not only helpful to distinguish the severity of angioedema and progressive necrosis but also helpful for the identification of pancreatic necrosis, chronic edema severity, and peripancreatic and extrapancreatic multipore exudate [17]. The morphological changes of pancreatic necrosis can be observed during contrast-enhanced CT examination, which is of great significance for judging the severity during examination; is also helpful for early detection, staging diagnosis of severity, and grading criteria; and can detect the presence of adverse complications. The qualitative and quantitative data analysis of pancreatic parenchyma and peripancreatic necrosis is also of significance for clinical diagnosis [18–20]. The general data of patients and the relationship between CTSI and PE involvement, RPS inflammatory infiltration, the number of peripancreatic effusion sites, and the degree of pancreatic necrosis examined by enhanced CT at different times were studied to explore the correlation between the degree and severity of CT inflammatory infiltration in RPS of AP and provide a reference for clinical treatment.

## 2. Materials and Methods

### 2.1. Study Subjects

From January 2021 to March 2022, 113 patients with AP were enrolled in the Department of Emergency Medicine of Anhui No. 2 Provincial People's Hospital. They were divided into groups according to CTSI classification, including 54 cases of grade I, 31 cases of grade II, and 28 cases of grade III. Clinical examination and laboratory data were obtained from the hospital. After the data were complete, enhanced CT detection was carried out in the hospital. The inclusion criteria and exclusion criteria are shown in Table 1. When the conclusions are released by using the patient's images and data, the individual privacy information of each patient is managed anonymously, ensuring the personal information security of each patient to the maximum extent. Before CT examination, patients knew the purpose, steps, and precautions of each examination, and in CT examination, the health status of each patient must be closely monitored to ensure the safety of the examination. It was approved by the Medical Ethics Committee of Anhui No. 2 Provincial People's Hospital. The patients and their families understood the content and methods and agreed to sign the corresponding informed consent form.

### 2.2. Diagnostic Criteria

The criteria for AP judgment in the 2012 Atlanta Global Cooperative Consensus are shown in Table 2.

At least two of the above criteria were met to confirm the diagnosis of AP. Criteria for moderate to SAP: transient organ failure (normal organ function within 48 hours) and/or local disease after onset. Criteria for SAP: persistent organ failure after onset (organ failure for more than 48 hours). Diagnostic criteria for organ failure were assessed using the revised Marshall score. Local complications included evaluation of the modified Marshall scoring system. Local diseases were mainly divided into acute peripancreatic effusion, acute necrotic aggregation, pseudocyst, capsular injury, pancreatic injury with infection, portal vein and hepatic vein thrombosis, acute gastric outflow obstruction, gastrointestinal fistula, abdominal bleeding, and PE.

“*2004 Chinese Guidelines for the Diagnosis and Treatment of Acute Pancreatitis* (Draft)”: the clinical manifestations of AP are acute persistent abdominal pain (no abdominal pain occasionally), elevated serum amylase activity 3 times above the upper limit of normal, imaging findings with or without pancreatic morphological changes, excluding other diseases. SAP was defined as one of the following criteria: organ failure (especially shock, pulmonary insufficiency, and renal failure); local complications (pancreatic necrosis, pseudocyst, and pancreatic abscess); Ranson score ≥3; APACHEii score ≥8; and grades *D* and *E* of CT.

### 2.3. Imaging Grading and Clinical Severity Grading Standard of AP

According to Balthazar grading, pancreatic Balthazar grading was divided into 5 grades (*A* ∼ *E*), with 0∼4 points in turn (Table 3).

The grading criteria (3 grades) for pancreatic necrosis were degree of necrosis <30%, 30% ∼ 50%, and >50%. Pancreatic necrosis and necrotic area accounted for 30% of the pancreas, Balthazar score plus 2 points; necrotic area accounted for 50% of the pancreas, Balthazar score plus 4 points; necrotic area accounted for more than 50% of the pancreas, Balthazar score plus 6 points.

CTSI = Balthazar AP grade + degree of pancreatic necrosis. CTSI divided AP into three different grades: grade I 0∼3 points, grade II 4∼6 points, and grade III 7∼10 points. CTSI >4 was classified as severe pancreatitis. The degree of inflammatory infiltration in the RPS was classified into four grades: grade *A*, without RPS involvement; grade *B*, with APS involvement only; grade *C*, with both APS and PS involvement; and grade *D*, with APS, PS, and PPS involvement.

### 2.4. Data Acquisition

CT examinations were performed using a 16-row (Somatom Sensation 16; Siemens Medical Solutions, Erlangen, Germany) or 64-row (GE Healthcare, Milwaukee, WI, USA) CT scanner with a display field of view (FOV) of 35 cm, tube voltage of 120 KV, tube current of 140 mA, and scanning range from the diaphragmatic surface of the liver to the pelvis. The contrast agent was 300 mg I/mL with Ultravist (Schering, Germany) or 300 mg I/mL with Iopamiron (Schering, Germany) or 300 mg I/mL with Omnipaqu (Nycomed, Norway), and the contrast medium was injected intravenously into the forearm with a high-pressure syringe at a dose of 80–100 mL. For further enhanced examination, a three-dimensional fat-saturated t1 weighted sequence was used for enhanced scanning. A gadolinium-based contrast agent (0.1 mmoL/kg) was injected with a high-pressure injector at a rate of 3–4 mL/sec, followed by 20 mL of normal saline. The injection rate was 2 mL/sec. Before the examination, the patients were required to actively cooperate during the examination and complete all sequences as much as possible. If the inspection process could not continue, the inspection was stopped. During the examination, the patients were required to lie flat, breathe as calmly as possible, and wear soundproof earplugs.

### 2.5. Statistical Processing

All statistical analyses were performed using IBM SPSS Statistics 26 software. Measurement data are expressed as the mean ± standard deviation. Comparisons were performed by *t*-test or analysis of variance. Statistical data were expressed by absolute logarithm and percentage, *χ*^2^ test was used for comparison, chi-square segmentation was used for pairwise comparison among three groups, rank sum test was used for comparison of rank data, and Spearman analysis was adopted for correlation analysis. Normally distributed quantitative data were evaluated using the Kolmogorov–Smirnov test, and variance alignment was evaluated using Levene's test. The quantitative data that met a normal distribution are expressed as the mean ± standard deviation ($\bar{\text{x}}$ ±*s*); the quantitative data that did not meet a normal distribution are expressed as the median and interquartile range. Qualitative data were expressed as percentages. Differences in quantitative data were compared by adopting Student's *T*-test or the Mann–Whitney *U* test. One-way variance (ANOVA) was applied to compare the quantitative data among the three groups, and Tukey's test was adopted for pairwise comparison. Qualitative data were compared using Pearson's *χ*^2^ test or Fisher's exact test. The measured fluid volume in each anatomical space in two rounds was observed (after the first round of CT measurement at admission, the same patient was measured again in the same order every other week). Data from both rounds were recorded using intraclass correlation coefficients to determine the reproducibility of the measured data.

## 3. Results

### 3.1. General Information

Of the 113 cases of AP, there were 54 patients with mild acute pancreatitis (MAP) and 59 patients with SAP. The CT images of MAP and SAP patients were randomly selected (Figure 1).

According to the general data, there were 75 males with a mean age of 47.45 ± 17.05 years and 38 females with a mean age of 53.6 ± 20.04 years. In AP, the number of male patients was more than that of females, approximately twice that of females, and the mean age of onset in females was later than that in males, and the difference was statistically significant (*P* < 0.01). The causes were biliary in 44 cases (39.0%), alcoholic in 20 cases (17.7%), hypertriglyceridemia (HTG) in 17 cases (15.0%), overeating in 29 cases (25.7%), other causes in 3 cases, accounting for 2.7%, and biliary as the main cause of AP (Figure 2).

### 3.2. Relationship between CTSI and Inflammatory Extension in the Retroperitoneum

To facilitate the statistics and analysis of subsequent data, AP patients were divided into three different grades according to CTSI, including 54 patients in grade I group, 31 patients in grade II group, and 28 patients in grade III group (Figure 3).

According to the classification of involvement: grade *A*, no RPS involvement; grade *B*, only APS involvement; grade *C*, both APS and PS involvement; and grade *D*, both APS, PS, and PPS involvement. Of the 113 patients, 62 had different degrees of RPS involvement, with a positive rate of 54.9% (62/113), and the overall involvement rates of APS, PS, and PPS were 46.9% (53/113), 53.1% (60/113), and 17.7% (20/113), respectively. APS involvement was predominant in grade I group; both APS and PS were predominant in grade II group, while APS, PS, and PPS were predominant in grade III group (Figure 4). PPS involvement in grade III group was greater than that in the grade I and II groups, and the difference was statistically significant (*P* < 0.05); that is, PPS involvement in the SAP group was higher than that in the MAP group.

In grade I group, inflammatory infiltration of RPS was mild, mainly grade *A* and *B*, accounting for 92.3% (49/54) and 7% (4/54), respectively; only 1 case of grade *C*, accounting for 1.9% (1/54), and no cases of grade *D*. In grade II group, the degree of inflammatory infiltration of RPS was mainly grade *C* in 87.1% (27/31), grade *B* and grade *D* in 3.2% (1/31) and 9.7% (3/31) of the cases, respectively. In the grade III group, the degree of infiltration was mostly above grade *C*, mainly grade *D*, accounting for 67.9% (19/28). The results of the correlation test showed that the difference was statistically significant (*P* < 0.01) (Figure 5). The degree of inflammatory infiltration in the RPS increased with increasing CTSI score (*P* < 0.05); that is, the more significant the inflammatory infiltration in the RPS, the more the severity of AP.

### 3.3. Relationship between CTSI and PE

In grade I group, 11 cases were complicated with PE in 54 cases, with a positive rate of 20.4%; in grade II group, 16 cases were complicated with PE in 31 cases, with a positive rate of 51.6%; in grade III group, 22 cases were complicated with PE in 28 cases, and the positive rate was 78.6%. Chi-square test among the three groups: the difference was statistically significant, *P* < 0.01; chi-square segmentation was used for pairwise comparison; grade I group was compared with grade II group, *P* < 0.01; grade I group was compared with grade III group, *P* < 0.05; grade II group was compared with grade III group, *P* < 0.05; the incidence of PE in grade I, II, and III groups was different, and the incidence of PE increased with the increase of CTSI score. The incidence of PE in SAP was higher than that in MAP, and the false line in Figure 6(a) indicates the positive and negative predictive curve. Nine cases of PE were found in AP patients with an onset less than 48 h, including four cases, four cases, and one case in the grade I, II, and III groups; PE was found in 40 AP patients with an onset more than 48 h, including 8 cases in grade I group, 11 cases in grade II group, and 21 cases in grade III group. The incidence of PE in the group greater than 48 h was higher than that in the group less than 48 h (*P* < 0.05), and the incidence of PE increased with increasing CTSI score. The above data are shown in Figure 6(b).

### 3.4. The Relationship between CTSI and the Number of Peripancreatic Effusion Sites

There were 76 cases (67.3%) of peripancreatic effusion, including 28 cases (51.9%) of peripancreatic effusion in the grade I group, 23 cases (74.2%) of peripancreatic effusion in the grade II group, and 25 cases (89.3%) of peripancreatic effusion in the grade III group. When there was 1 effusion, the grade I group accounted for the highest proportion (34.7%), while having ≥2 effusions. The proportion gradually increased with disease aggravation. In conclusion, when the disease severity increased, the number of peripancreatic effusion sites increased, and the difference was statistically significant (*P* < 0.01). The correlation analysis results with the disease severity showed that there was a positive correlation between the two (*P* < 0.01). The distribution of the number of peripancreatic effusion sites in each group is shown in Figure 7.

### 3.5. Grading of pancreatic necrosis by enhanced CT at different times

Grades I, II, and III of the CTSI grade correspond to three grades of the degree of pancreatic necrosis: necrosis <30% grade, 30% < necrosis <50% grade, and necrosis >50% grade, respectively. Contrast-enhanced CT 1 ∼ 2 days after onset in AP patients showed that pancreatic necrosis was mainly necrosis <30% grade, accounting for 27.8%, and necrosis >50% grade accounted for 7.1%. 3 ∼ 4 days after onset, pancreatic necrosis was mainly 30% < necrosis <50% grade, accounting for 38.7%, and necrosis >50% grade accounted for 25.0%. 5 ∼ 6 days after onset, pancreatic necrosis was mainly necrosis >50% grade, accounting for 42.9%; 7 ∼ 8 days after onset, pancreatic necrosis was mainly necrosis <30% grade, accounting for 16.7%, and necrosis >50% grade accounted for 10.7%. More than 8 days, necrosis <30% grade, 30% < necrosis <50% grade, and necrosis >50% grade accounted for 14.8%, 12.9%, and 14.3%; the detection rate of necrosis >50% grade found by enhanced CT 5 ∼ 6 days after onset was higher than other time periods (*P* < 0.05), indicating that pancreatic necrosis was more likely to be found by enhanced CT 5 ∼ 6 days after onset (Figure 8).

## 4. Discussion

AP is a common acute abdomen in clinical treatment, often involving many organs of the body. Its disease complications are very strict, and the mortality rate is high. It is clinically divided into acute MAP and SAP. SAP accounts for about 20% of AP. The clinical pathological changes during treatment are very complex, with a mortality rate as high as 2/10–3/10. Timely and correct evaluation of the severity of AP and reasonable systematic treatment will help to improve the prognosis of patients [21]. Ultrasonography can also be the most important detection modality for AP imaging, but because the results of ultrasonography are susceptible to gastrointestinal air accumulation, while CT examination can reveal significant changes in the morphology and pathology of AP, CT examination is also the most accurate imaging modality for the detection of AP, and enhanced CT examination is helpful to identify the severity of necrosis and chronic edema in the pancreas and the status of peripancreatic and extrapancreatic multiple space exudates [22]. As medical care progresses, multiple assessment systems have been developed.

The RPS is defined as having three spaces: PS, APS, and PPS. The PS consists of the anterior renal fascia on the front of the kidney and the posterior renal fascia on the back. Bridging septa composed of connective tissue are widespread in the PS fat, between the renal capsule and the renal tendon layer, between the anterior and posterior renal muscle layer, and between the renal capsule and capsule [23, 24]. Most researchers proposed to continue to spread AP to the RPS, including the pancreatic enzyme exudate rich in AP, because histolytic effect can cause the melting of the renal muscle layer and cause inflammatory edema and effusion between the renal tendon layers. When the inflammation exceeds the prerenal and retrorenal muscle layers, the inflammation continues to proliferate and infiltrate APS, PS, PPS, etc., and cause transmuscular and trans-space spread of retroperitoneal changes. When effusion occurs in PPS, the mortality rate of AP patients is increased, while when examination shows PPS involvement, the risk of SAP is great, so PPS involvement can also be used as an important indicator for the diagnosis of SAP. If PPS involvement is used as a positive criterion for judging SAP, its specificity (88.2%) and positive predictive value (91.8%) indicate that after PPS involvement, the risk of working for SAP is greater, but it generally does not affect MAP judgment [25–27]. APS involvement was more common in MAP, while both APS and PPS involvement were more common in SAP. The degree of inflammatory cell infiltration in the retroperitoneum could reflect the severity of AP to some extent. Particularly, the involved period of PPS mostly is shown as SAP, so the disease can be managed as SAP during the involved period of PPS.

Patients with AP are more likely to have confluent lung disease, including human PE, atelectasis, lung disease, or concurrent ARDS and circulatory depletion. There are many studies on PE in China. At present, it mainly holds the view that peripancreatic inflammation spreads from the extrapancreatic to the pleural cavity to form PE [28]. It is generally believed that anatomically, the lymphatic plexus around the transverse septum is connected with the mediastinal and subcostal spaces, the giant inflammatory cells formed by AP spread into the mediastinum and subcostal space through the lymph plexus around the septum, and the pancreatic enzyme effusion containing soluble tissue gradually entered the chest cavity. PE is important for assessing the severity and prognosis of AP and is the main symptom of extrapancreatic involvement of AP [29]. Although PE can also be detected radiologically early, most of them occur earlier than the date of pancreatic injury, and the incidence of PE increases with increasing CTSI score [30]. This revealed that PE can be recommended as a reference technical index for the diagnosis of severe pancreatitis, especially if PE is found within 24 hours after onset, and the mortality rate will be significantly improved. It was also found that there was a difference between PE and the incidence in patients with MAP/SAP, and if the incidence of AP patients with PE was more severe in early detection, it could also be used as an early index for AP severity judgment.

Early contrast-enhanced CT examination without significant changes is often found in clinical practice in pancreatic necrosis, and a second contrast-enhanced CT examination can detect massive pancreatic necrosis. Patients with early pancreatitis had CTSI scores of grades I and II, and over time, patients developed grade III. This is because it takes some time for the inflammation of the pancreas to transform into necrosis, and it also takes some time for imaging changes. It should be noted that there is a time difference between the imaging findings of AP and the clinical presentation. If CT enhancement is performed early in patients with AP, some SAP may be misdiagnosed as MAP. Therefore, the optimal time for AP-enhanced CT examination can be better used for the corresponding treatment [31, 32]. Many clinical data have demonstrated that changes in pancreatitis can be found by CT 12 h-24 h after onset, but there is no uniform consensus on the time of contrast-enhanced CT examination. Enhanced CT 2–3 days after admission more easily distinguishes interstitial pancreatitis from necrotizing pancreatitis than enhanced CT on admission [33]. Since pancreatic necrosis does not occur early, some studies suggest that SAP is dynamically enhanced 3–0 days after admission to avoid affecting the early assessment of disease severity by CTSI.

A total of 113 patients with AP were retrospectively analyzed. If pancreatic necrosis occurs 5–6 days after the onset of the disease detected by enhanced CT, it can be found to the maximum extent, but it is not the peak period of AP severity. The imaging causes of AP: the imaging findings of AP have a certain time difference compared with the clinical manifestations. It takes a certain time for exudative inflammation of the pancreas to develop into pancreatic necrosis, which is a pathological change, and it also takes a certain time for the corresponding changes to be found by imaging monitoring. According to the principle of enhanced CT imaging, when the normal pancreatic tissue progresses to the completion of pancreatic liquefaction necrosis, the enhanced contrast agent cannot be perfused into the necrotic pancreatic tissue through the microcirculation, and the pancreatic parenchymal necrosis shows an unenhanced low-density pancreatic area on imaging.

## 5. Conclusion

The examination of the degree of retroperitoneal inflammatory infiltration showed that the higher the degree of inflammatory infiltration was, the higher the severity of AP was. Especially when PPS is involved, SAP is often recommended. Therefore, when PPS is involved, the patient's condition can be treated according to SAP. Analysis of AP patients with early PE found that the condition of AP patients with PE was more serious, and PE can be used as an early indicator of AP severity. According to the analysis of the degree of pancreatic necrosis in AP patients, the maximum range of pancreatic necrosis can be found by enhanced CT examination 5–6 days after the onset of AP.

## Figures and Tables

**Figure 1:** Example of the severity grade of AP. (a) and (b) are MAP, patchy low-density nonenhanced areas; (c) and (d) are SAP, and large patchy effusion shadows are observed.

**Figure 2:** General data of patients. (a) Gender ratio of the two groups, (b) Etiological comparison of the two groups, in which ^∗∗^ represents the difference with statistical significance (*P* < 0.01).

**Figure 3:** CTSI grouping of patients with AP.

**Figure 4:** CTSI classification and RPS involvement. (a) Number of involvements, (b) Involvement of different grades; ^∗^indicates that the difference is statistically significant (*P* < 0.05).

**Figure 5:** CTSI grading and degree of inflammatory infiltration in RPS. (a) Number of cases with different degrees of infiltration, (b) Proportion of cases with different degrees of infiltration; ^∗^represents the difference with statistical significance (*P* < 0.05), ^∗∗^represents the difference with statistical significance (*P* < 0.01).

**Figure 6:** Relationship between different CTSI groups and PE. (a) Detection rate of PE of different CTSI grades (in grade II group, ^#^ represents comparison with grade I group, in grade III group, ^#^represents comparison with grade I group and grade II group, respectively); (b) Number of PE cases at different time points; ^∗^represents the difference has statistical significance (*P* < 0.05), ^∗∗^represents the difference has statistical significance (*P* < 0.01), ^#^represents comparison among groups (*P* < 0.05), ^##^represents the difference has statistical significance (*P* < 0.01).

**Figure 7:** Distribution of the number of peripancreatic effusion sites in each group. ^*∗*^indicates a statistically significant difference (*P* < 0.05), and ^*∗∗*^indicates a statistically significant difference (*P* < 0.01).

**Figure 8:** Degree of pancreatic necrosis at different time periods. ^*∗*^represents a statistically significant difference (*P* < 0.05).

**Table 1:** Inclusion criteria and exclusion criteria of study subjects.

Serial number	Inclusion criteria
1	Diagnostic criteria in line with AP
2	Enhanced CT examination after admission
3	Inpatients with complete clinical and laboratory data

	Exclusion criteria
1	Patients with severe primary diseases in cardiovascular, liver, kidney, or hematopoietic system
2	Age <18 years old
3	AP caused by trauma, surgery, and tumor
4	Patient being unable to stop consciousness due to agitation and involuntary movement

**Table 2:** Judgment criteria for AP.

Serial number	Judgment criteria
1	Acute abdomen such as upper abdominal pain and discomfort
2	Serum lipase or amylase level 3 times or more above the normal upper limit
3	CT imaging of the abdomen suggesting the diagnosis of AP

**Table 3:** Balthazar grading of the pancreas.

Grade	Content	Point
*A*	Normal pancreas	0
*B*	Diffuse or focal pancreatic enlargement, including irregular contour, uneven density, pancreatic duct dilatation, small hydrops in the gland, without peripancreatic changes	1
*C*	Abnormalities in vivo associated with inflammatory changes in peripancreatic adipose tissue characterized by peripancreatic blurring and strip density	2
*D*	Single effusion focus or honeycomb inflammatory mass with unclear boundary	3
*E*	Having two or more effusions or pneumatosis with unclear boundary in glands or adjacent areas	4

## Data Availability

The datasets used and/or analyzed during the current study are available from the corresponding author upon reasonable request.
